The article "Effect of Application of Different Exercise Intensities on Vitamin D and Parathormone in Children with Down's Syndrome" was retracted in 2023. Reasons: signs of a paper mill; compromised peer review; unreliable results or conclusions.

# Effect of Application of Different Exercise Intensities on Vitamin D and Parathormone in Children with Down's Syndrome

**DOI:** 10.1155/2021/7424857

**Published:** 2021-12-07

**Authors:** Hatem H. Allam, Alaa Shafie, Amal F. Gharib, Ahmad El Askary, Mazen Almehmadi, Tarek Alsayad, Ahmed M. Alziyadi, Lamiaa K. Elsayyad

**Affiliations:** ^1^Physical Therapy Department, College of Applied Medical Sciences, Taif University, Saudi Arabia; ^2^Department of Clinical Laboratory Sciences, College of Applied Medical Sciences, Taif University, P.O. Box 11099, Taif 21944, Saudi Arabia; ^3^Lecturer of Pediatrics, Faculty of Medicine, Al-Azhar University, Cairo, Egypt; ^4^Academic Affairs Director, Prince Sultan Hospital, Taif, Saudi Arabia

## Abstract

**Background:**

Children with Down's syndrome are more liable to vitamin D deficiency. Treating this deficiency with supplements is associated with the risk of intoxication.

**Aim:**

The study is aimed at comparing the effect of two exercise intensities on the modulation of vitamin D and parathormone levels in children with DS.

**Methods:**

Forty-four DS male children aged from 8 to 12 years participated in the study. They were assigned randomly into two equal groups. Group I received high-intensity treadmill aerobic exercises, and group II received moderate-intensity T-AE, three times per week for three months. The blood samples were collected from both groups before the intervention, after one month of intervention, then after three months of intervention to assess serum 25(OH)D and PTH levels.

**Results:**

Repeated measure MANOVA revealed that the high-intensity T-AE induced a significant increase in 25(OH)D after one month and after three months while it significantly decreased PTH only after three months. Moderate-intensity T-AE had a nonsignificant effect on both hormones.

**Conclusion:**

The current study concluded that the high-intensity T-AE improved both vitamin D and parathormone serum levels after three months of intervention.

## 1. Introduction

Down's syndrome (DS) is the commonest chromosomal disorder that causes mental retardation. It occurs in 1 in 700–1000 live births [1]. Also, they suffer from certain medical disorders like congenital heart disease, visual and auditory problems, immune and endocrinal problems, and orthopedic problems as reduced muscle tone and strength and laxity of their ligaments [2].

The normal level of 25(OH)D is very important because it may assist in protection against certain diseases as diabetes mellitus type 1, hypertension, and the development of cancer [3]. Moreover, vitamin D was found to be an important factor in psychological human health [4]. Additionally, it was noticed that vitamin D deficiency is a common health problem even among children of sunshiny areas such as Jeddah, Kingdom of Saudi Arabia, which is associated with health problems such as rickets. The deficiency may be related to certain factors as malnutrition or decreased physical activity level [4]. Vitamin D level is detected by serum 25(OH)D levels, which are categorized as the following: ≤10 ng/mL (severe deficiency), 11–20 ng/mL (deficiency), 21–30 ng/mL (insufficiency), and >30 ng/mL (sufficiency) [5].

Elsayyad et al. [6] added that the Vit D and PTH levels are related to physical performance. The skeletal muscles and their activities play a critical role in the metabolism of Vit D and PTH levels. Additionally, Aly et al. [7] reported that moderate-intensity swimming exercises improved Vit D status in rats with induced type II diabetes. On the other hand, lack of sports and physical activity is accompanied by decreased serum calcium or 25(OH)D [8]. Vitamin D plays a very important role in Down's syndrome children's health. Vitamin D status differs widely between different nations. This depends on several factors such as dissimilar exposures to sunlight, Vit D supplementation, physical activity levels, and dietary intake of vitamin D [9].

Stagi et al. [10] reported that there was a Vit D deficiency and high PTH levels in children with DS so it is serious to evaluate its levels in these subjects. The decreased 25(OH)D levels may be also due to reduced dietary intake and physical activity levels. Treating this deficiency with Vit D supplements may be associated with the risk of Vit D intoxication due to increased intestinal absorption or decreased vitamin D metabolism [11]. So, the study is aimed at comparing the effect of two exercise intensities on the modulation of serum vitamin D and parathormone (PTH) levels in children with DS.

## 2. Materials and Methods

### 2.1. Study Design

A randomized controlled trial was used to investigate the effect of application of two exercise intensities on vitamin D and PTH levels in children with Down's syndrome. The study was conducted at the College of Applied Medical Sciences. All participants have undergone the initial clinical examination by the same examiner at the beginning of the study. The study was double-blinded, and both the examiners and participants were blinded about the group division. The enrolment of the participants was done by telephone calls to their parents or legal guardians to explain the nature and value of the study. We conducted interviews with the parents and their sons to take the demographic data, clarify to them the steps of the study, let them sign the written consent form, and take the medical history, periods of sun exposure, and food frequency questionnaire (FFQ).

### 2.2. Subjects

A total of fifty male DS subjects were initially selected to participate in the study. Only forty-four subjects completed the interventional study because six children were excluded (Figure 1). Their age was ranged from 8 to 12 years. The participants were assigned randomly using sealed envelopes into two equal groups; group I (GI) and group II (GII) each contain twenty-two subjects. GI received the high-intensity T-AE, and the GII received the moderate-intensity T-AE, three times per week for three months. The simple randomization technique was used. All subjects were selected from children's hospitals at the Western area, Saudi Arabia.

### 2.3. The Inclusion Criteria

All subjects were able to walk freely without assistance. They had vitamin D deficiency, and the serum level of 25-hydroxyvitamin D (25(OH)D) was ranged from 10 to 20ng/mL [5]. Additionally, they did not take calcium or vitamin D3 supplements, medications for osteoporosis, antiepileptic drugs, or any medications that may affect the Vit D metabolism in the last 5 months. The feeding method during the first two years of age for all children was bottle feeding. Their IQ ranged from 45 to 70 to be able to understand simple orders. They were free from any medical consequences, for example, auditory defects and visual impairments. Besides, they had no previous history of strength training. Their body mass index percentile ranged from the 50th percentile to less than the 75th percentile (healthy).

### 2.4. The Exclusion Criteria

The participants were excluded if they had an autoimmune disease and renal diseases, have taken any thyroid medications, are suffering from obesity and epileptic fits, or had a BMI percentile above 75th or below 50th. All participants had received an agreement from their medical doctor before enrolment in the study. A flowchart showing the children who participated in the study is illustrated in Figure 1.

### 2.5. Anthropometric Parameters

Body mass index percentile was utilized as an assessment method to ensure that all children were categorized as healthy. A Seca digital scale (Seca model 770, made in Germany) and a calibrated measuring rod (Seca Road Rod) were used to measure the children's weight and height. The body weight and standing height were measured while the child in bare feet with minimal clothing three times to reduce the faults. Body mass index (BMI) was calculated by dividing the weight (kg) by height (m) squared. The BMI percentile then was calculated from the recommended charts to categorize each member.

### 2.6. Intelligence Quotient (IQ) Level

A clinical psychologist used the Binet Kamat test which is the Indian version of the 1934 version of the Stanford–Binet scale and has been used to determine the IQ level [12].

### 2.7. Dietary Intake and Sun Exposure

Calcium and vitamin D intake in the diet was assessed by interviews with the parents. Saudi (FFQ) was used. It is a modified form of food frequency questionnaire established by the European Prospective Investigation into Cancer and Nutrition (EPIC) study. It includes the food elements that frequently eaten by the Saudi residents [13]. The parents recorded the types and the amount of the consumed food for every meal for their children daily for one week. The FETA computer program was used to analyze the obtained data from the FFQ [14]. The sun exposure was calculated as the number of hours/weeks expended outdoor registered by the parents.

### 2.8. Physical Activity

The physical activity questionnaire adapted from Baecke et al. [15] was used to assess the participants' physical activity level. The scores of both sports and leisure time were detected by this questionnaire. Both values were summed to give the total physical activity score. The physical activity score was ranged from 4 to 7. All participants who had a physical activity score of less than 4 or more than 7 were excluded.

### 2.9. Blood Measurements

The blood analysis was done at three points, at the beginning of the study, after one month of intervention, and after three months of intervention at the same time from the day (at 9 AM). Blood samples were obtained from all participants after 10-hour overnight fast. Five cubic centimetres of blood was drawn. The serum level of parathormone (PTH) and 25(OH)D was detected using enzyme-linked immunosorbent assay (ELISA) test. It is a simple, fast, and reliable technique, so it has been developed and improved for detecting organic constituents of biological fluids including blood because.

### 2.10. Calculation of Exercise Intensity

We used the Martti Karvonen formula to calculate the heart rate zone. Firstly, the resting heart rate (rest-HR) was detected for every participant by inviting him to lie in a prone position for 10 minutes while catching a heart rate monitor. After that, the maximum heart rate (max-HR) was calculated by utilizing this formula: maximum heart rate = 220 − age. Then, we calculated the heart rate reserve (HRR) by using the law: HRR = max − HR–resting HR. Exercise intensity is represented as a percentage of HRR. Finally, the target heart rate (target-HR) was calculated by using the formula: target − HR = HRR × intensity% + rest − HR. The moderate-intensity exercises were defined as the activity which uses 50% to 70% of the HRR, while the high-intensity exercises use 70% to 90% of the HRR [16].

### 2.11. The Intervention

All participants were asked to present at the rehabilitation unit at the same time of the day. They were asked to come to the rehabilitation unit three days before the intervention and try all intervention procedures to be more familiarized. GI received high-intensity T-AE while GII received moderate-intensity T-AE, three times per week, for three months using a motorized treadmill [17]. Each participant started the training session with 5-minute warm-up in the form of running in place and finished it with 5-minute cooldown in the form of gentle stretching exercises for lower limb muscles, with twenty seconds for stretching followed by twenty seconds for relaxation. The intervention for both groups was done as shown in Table 1. The inclination was 5° up. The speed of the treadmill started by 2.5 mills/hour then gradually increased by 0.5 mills/h every 5 minutes until the target heart rate reached. Participants had been permitted to use the handrails according to the need. To ensure regularity in attending the training program, we have taken the participants' attendance in all sessions.

### 2.12. Ethical Considerations

The study was conducted according to the guidelines of the Declaration of Helsinki and approved from the Research Ethics Committee, Taif University, Saudi Arabia (approval number 42-0010), and the ethical committee at the Research and Studies Department, Directorate of Health Affairs, Taif, Saudi Arabia (IBR Registration number with KACST, KSA HAP-02-T-067) (approval number, 428).

### 2.13. Statistical Analysis

A pretest power analysis (power, 0.80; *α* = 0.05; effect sizes = 0.5, Pillai V = 0.2) was used to detect the sample size for this study. SPSS version 26 was used for statistical analysis. Shapiro-Wilk test (*P* > 0.05), Q-Q plots, skewness, and kurtosis were used to ensure that the data were near the normal distribution. Levene's test and Box's test showed nonsignificant values (*P* > 0.05). Repeated measure MANOVA test and Bonferroni pairwise comparisons were used to declare within and between subjects' differences in the serum levels of both hormones before and after the intervention.

## 3. Results

### 3.1. Demographic Data

There were no significant differences between the two groups regarding the mean of sun exposure and vitamin D intake during the study period, age, BMI percentile, or physical activity level.  Table 2 illustrates MANOVA results and Bonferroni pairwise comparisons of the demographic data.

### 3.2. Study Variables

According to the study variables, we could not assume sphericity using Mauchly's test or Greenhouse-Geisser correction, so we used Huynh-Feldt for sphericity correction. Regarding Box's test (*P* > 0.05) and Levene's test (*P* > 0.05), they indicated equality of covariance and equality of variance between the two groups, respectively.  Table 3 demonstrates repeated measure MANOVA within subjects' effects and between subjects' effects.

### 3.3. Vitamin D Level (ng/ml) and PTH Level (pmol/L)

Regarding vitamin D levels, high-intensity exercises led to a significant increase in vitamin D levels after one month of the intervention when we compared it to its basal level. After three months of the intervention, GI showed a significant increase in Vit D when compared to its level in GII and to its basal level. There was a nonsignificant increase in serum Vit D level in GII after one month and after three months of the intervention (Table 4). Pairwise comparisons showed a significant decrease in PTH level in GI at the endpoint when compared to its basal level and to the PTH level of GII at the endpoint. After one month of intervention, PTH level in GI showed a nonsignificant decrease when we compared it to its basal level or to its level in GII. Regarding GII, the decrease in the PTH level was nonsignificant after one month or after three months of intervention when it was compared to its basal level (Table 5).

## 4. Discussion

The study is aimed at investigating the effect of two different exercise intensities on vitamin D and parathormone levels in children with Down's syndrome. We have selected the children with DS as Stagi et al. [10] and Zubillaga et al. [18] mentioned that they have Vit D deficiency and hyperparathyroidism. This comes in agreement with our basal analysis of both hormones at the beginning of the study. It was crucial to study Vit D and PTH in combination with each other because there is a high relation between them. Vit D itself is not an active element as it needs to be transformed into the active form of Vit D in the liver and kidney, and this process requires the presence of PTH [19].

Concerning the effect of moderate and high-intensity exercise programs on Vit D, the results of the study revealed that there was a significant increase in Vit D level in GI after application of the high-intensity exercise program at both midpoint and endpoint compared with its basal concentrations. These findings are confirmed by Kluczynski et al. [20], who reported that there was a higher level of 25(OH)D concentration due to the application of higher-intensity regular exercises and physical activity, and this relationship was maintained even after sun exposure adjustment. Lanteri et al. [21] added that muscle-strengthening exercise is associated with improved serum 1,25(OH)2D3 levels. According to Mason et al. [22], the muscle tissue serves as important storage of 25(OH)D and returns it to the circulating blood when required. They added that the muscle provides a significant site of sequestration of 25(OH)D, protecting it from degradation in the liver. This could explain why training, not only outdoors, is related to better vitamin D status. In contrast, Maimoun et al. [23] contradict our findings as they mentioned that the serum 25(OH)D level did not change after maximum incremental exercises. However, in this study, the participants performed a maximum incremental exercise test not a training regimen and the blood samples were collected immediately after the exercise. Over and above that, Iwamoto et al. [24] confirmed our results when they mentioned that eleven weeks of high-intensity treadmill exercise increased the serum 1,25-dihydroxyvitamin D3 level and increased intestinal absorption of calcium. They related the vitamin D elevation to the treadmill exercises stimulated bone formation and suppressed bone resorption, resulting in high demand for minerals that were satisfied by the increased level of the serum 1,25-dihydroxyvitamin D3 and increased intestinal absorption of calcium. Furthermore, Vainionpää et al. [25] coincided with our findings as they reported that serum basal 25(OH)D increased significantly after the application of high-impact exercises three times per week for 6 months. Moreover, Maimoun et al. [26] reported that a single session of strenuous exercises elevated serum 25-hydroxyvitamin D which supported our results.

Additionally, Barker et al. [27] come in agreement with us when they mentioned that the serum 25(OH)D concentrations were significantly increased after the application of a high-intensity exercise program on a group of young adults. They attributed this increased level of 25(OH)D to the elevation in albumin concentrations circulating in the blood. Additionally, Sun et al. [28] mentioned that the serum 25(OH)D concentrations were significantly increased after application of high resistance training exercise program for 12 weeks at both midpoint and endpoint in comparison with baseline values. According to Makanae et al. [29], the increased level of serum 25(OH)D may be also attributed to the significant increase in intramuscular CYP27B1 after the application of high-intensity exercises that catalyzes the hydroxylation and activation of 25(OH)D, which may boost local vitamin D metabolism in skeletal muscles.

Concerning the PTH serum level, the results of the study revealed that there was a significant decrease in PTH level in GI after three months of high-intensity exercises when compared to its basal level and to the PTH level of GII after the intervention. Vainionpää et al. [25] agreed with our findings as they reported that the serum basal PTH decreased significantly after application of high-impact exercises, three times per week. They related this decline in serum PTH to changes in vitamin D metabolism which have an inverse relation with serum PTH concentration according to Ardehali et al. [30]. Additionally, Scott et al. [31] supported our results as they reported that the serum PTH concentration was only transiently increased immediately after conducting an exercise program with 75% VO2 max and was decreased from the basal value at 4 days after the endpoint. Sun et al. [32] come in consistency with our findings when they mentioned that the PTH concentrations were transiently increased and then reduced after application of a cycling exercise for 30 minutes at 70% maximal oxygen uptake.

Additionally, Iwamoto et al. [24] supported our results when they reported that the high-intensity treadmill exercises decreased serum PTH level due to increased calcium absorption which suppressed the serum PTH level. Furthermore, the decreased PTH concentration may be related to increasing physical fitness after application of high-intensity exercises; this is according to Brahm et al. [33], who reported that there was an inverse relationship between physical fitness and PTH serum level. They added that the high physical fitness and active long-term endurance training have been accompanying a decreased basal PTH levels.

On the other hand, Barry and Kohrt [34] contradicted our results when they conducted a study to investigate the effects of a 2-hour exercise bout at controlled workloads of 75% of the ventilatory threshold on calcium and serum PTH level in 20 competitive male cyclists. They found that the PTH concentration was increased immediately after the application of the exercise session. This contradiction may be related to the following: firstly, they studied the short-term effect of exercises on PTH; secondly, they studied the effect of one session training which differed from our exercise program. Additionally, Thorsen et al. [35] supported our results when they mentioned that the PTH serum level was not significantly affected by moderate endurance exercise. They mentioned that the intensity of the performed physical exercises was inadequate to significantly affect the PTH level.

### 4.1. Limitations

Firstly, only male children were selected to participate in the study without having female participants because of cultural values in Saudi Arabia. Secondly, certain biomarkers related to vitamin D, such as calcium, and phosphorus levels were not analyzed and could contribute to the relationship between exercise performance and vitamin D.

## 5. Conclusions

The high-intensity treadmill aerobic exercises had a significant influence on the serum vitamin D and parathormone levels while these hormones were not significantly affected by the moderate-intensity aerobic exercises.

## Figures and Tables

**Figure 1:** Flowchart showing the children who participated in the study.

**Table 1:** The sequence of treadmill aerobic exercises (T-AE) for GI and GII.

Week	High intensity	Moderate intensity	Time (min)
1, 2	70%	50%	20
3, 4	75%	55%	25
5, 6	80%	60%	30
7, 8	85%	65%	35
9, 10	90%	67%	40
11, 12	90%	67%	40

**(a):** 

Multivariate test					
	Value	*F*	Hypothesis df	Error df	Sig.
Wilks' lambda	.912	.731	5.000	38.000	.604

**(b):** 

Bonferroni pairwise comparisons				
Demographic variables	GI M ± SD	GII M ± SD	MD (GI-GII)	Sig.
Sun (h/week)	15.68 ± 3.85	16.32 ± 3.06	-.64	.547
Vit D intake (mg/day)	104.86 ± 13.93	103.41 ± 14.9	1.46	.740
Age (year)	10.27 ± 1.45	10.18 ± 1.47	.091	.837
PA	4.91 ± .92	5.45 ± .91	-.55	.055
BMI percentile	69.50 ± 5.93	69.09 ± 6.04	.41	.822

M: mean; SD: standard deviation; MD: mean difference; PA: physical activity; BMI: body mass index.

**(a):** 

Tests of within subjects' effects (multivariate)						
Source	Test	Value	*F*	Hypothesis df	Error df	Sig.
Hormonal level	Wilks' lambda	.604	11.892	4.000	166.000	.000
Hormonal level ^∗^ group	Wilks' lambda	.885	2.607	4.000	166.000	.038

**(b):** 

Tests of within subjects' effects (univariate)							
Source	Measure	Test	Type III sum of squares	df	Mean square	*F*	Sig.
Hormonal level	PTH	Huynh-Feldt	1988.33	1.83	1086.47	14.43	.000
	Vit D		590.76	2.00	295.38	11.49	.000
Hormonal level ^∗^ group	PTH	Huynh-Feldt	525.46	1.83	287.12	3.815	.030
	Vit D		72.02	2.00	36.01	1.401	.252

**(c):** 

Tests of between subjects' effects						
Source	Measure	Type III sum of squares	df	Mean square	*F*	Sig.
Group	PTH	11.422	1	11.422	.156	.695
	Vit D	236.189	1	236.189	8.955	.005

PTH: parathormone; Sig.: significance; df: degree of freedom.

**Table 4:** Bonferroni pairwise comparisons for Vit D (within subjects and between subjects).

	Vit D ng/ml (M ± SD)			MD (within subjects)			
	Pre	Post1	Post2	Prepost1	Sig.	Prepost2	Sig.
GI	17.74 ± 5.38	22.72 ± 4.67	24.47 ± 4.29	-4.98	.013^∗^	-6.732	.000^∗^
GII	17.05 ± 5.26	19.62 ± 6.59	20.24 ± 3.93	-2.575	.383	-3.189	.082
MD (between subjects) GI-GII	.691	3.1	4.24				
Sig.	.669	.079	.001^∗^				

M: mean; SD: standard deviation; MD: mean difference. ^∗^Significant difference.

**Table 5:** Bonferroni pairwise comparisons for PTH (within subjects and between subjects).

	PTH pmol/L (M ± SD)			MD (within subjects)			
	Pre	Post1	Post2	Prepost1	Sig.	Prepost2	Sig.
GI	50.96 ± 9.08	46.82 ± 9.29	37.40 ± 9.18	4.14	.396	13.56	.000^∗^
GII	49.07 ± 9.40	44.25 ± 6.23	43.62 ± 6.41	4.82	.244	5.45	.171
MD (between subjects) GI-GII	1.89	2.56	-6.22				
Sig.	.501	.289	.013^∗^				

M: mean; SD: standard deviation; MD: mean difference. ^∗^Significant difference.

## Data Availability

The data used to support the findings of this study are available from the corresponding author upon request.
